# Porcine-Stimulated Human Tr1 Cells Showed Enhanced Suppression in Xenoantigen Stimulation Response

This article has been retracted.

**DOI:** 10.1155/2021/2725799

**Published:** 2021-11-08

**Authors:** Xiaoting Chen, Hongwen Ma, Lina Gong, Guang Yang, Xi Jin

**Affiliations:** ^1^Department of Urology, Institute of Urology, West China Hospital, Sichuan University, Chengdu, China; ^2^Animal Experimental Center, West China Hospital, Sichuan University, Chengdu, China

## Abstract

Type 1 regulatory T (Tr1) cells play a fundamental role in maintaining and inducing immune tolerance. Our preliminary study demonstrated that an interleukin- (IL-) 10-mediated pathway is a possible regulatory mechanism underlying the xenoantigen-specific human Treg enhanced suppressive capacity. Here, we developed a feasible protocol for expanding IL-10-induced xenoantigen-specific human Tr1 cells in vitro which would be more efficient in transplantation immunotherapy efficiency. In this study, xenoantigen-specific Tr1 cells are generated from human naive CD4^+^ T cells expanded for two subsequent xenoantigen-stimulation cycles with recombinant human IL-10. The phenotype and suppressive capacity of xenoantigen-stimulated Tr1 cells are assessed, and the mechanism of their suppression is studied. Tr1 cells can be induced by porcine xenoantigen stimulation combined with IL-10, IL-2, and IL-15, displaying an increased expression of CD49b, CTLA-4, and LAG-3 without expressing Foxp3 which also showed an effector memory Treg phenotype and expressed high levels of CD39. After xenoantigen stimulation, the IL-10 and IL-5 gene expression in Tr1 cells increased, secreting more IL-10, and xenoantigen-stimulated Tr1 cells changed their T cell receptor (TCR) V*β* repertoire, increasing the expression of TCR V*β*2, TCR V*β*9, and TCR V*β*13. In a pig to human mixed lymphocyte reaction (MLR), xenoantigen-stimulated Tr1 cells displayed enhanced suppressive capacity via CD39 in a dose-dependent manner. Moreover, IL-5 could affect the proliferation of xenoantigen-specific Tr1 cells, but not their phenotypes' expression. This study provides a theory and feasible method for immune tolerance induction in clinical xenotransplantation.

## 1. Introduction

Regulatory T cells (Tregs) are known to restrain immune responses to self-antigens, nonself-antigens, and associated inflammation [1]. Previous studies indicated that Tregs' adoptive transfer is an immunomodulatory therapy to prevent type 1 diabetes, autoimmune diseases, graft-versus-host disease (GVHD), and rejection during organ transplantation [2, 3]. Recently, accumulated evidence indicated that adoptive transfer with antigen-specific Tregs prevents xenograft rejection by downregulating the immune responses of effector T cells [3, 4] and tissue injuries by exerting on-targeted suppression function [5].

Type 1 regulatory T (Tr1) cells, a major class of Tregs, are characterized by the secretion of high levels of interleukin- (IL-) 10 and the coexpression of surface markers LAG-3 and CD49b without constitutive expression of FOXP3 and CD25, which have immune-suppressive potency and bear alloantigen specificity [6, 7]. Tr1 cells predominantly present high expression of TGF-*β* and low levels of IL-2, whereas the IL-5 and interferon- (IFN-) *γ* levels in Tr1 cells depend on the conditions [8]. IL-10 can control the differentiation and proliferation of Tregs and maintain peripheral T cell tolerance [9]. Previous studies showed that IL-10 positively affects the differentiation of Tr1 cells with regulatory functions from the peripheral blood mononuclear cell (PBMC) or CD4^+^ T cell after a long-term polyclonal or allospecific stimulation [10]. Extensive studies demonstrated that Tr1 cells, which represent the major subset of the regulatory T cell population, can reverse tissue damage and transplant survival in GVHD [11–13] and slow the progression of type 1 diabetes [14, 15]. Studies in transplantation animal models and clinical trials demonstrate that alloantigen-specific Tregs have superior antigen-specific efficacy compared with polyclonally exposed Tregs and can achieve targeted suppression and prevent allograft tissue, thereby reducing the risk in transplantation [14, 16–18]. However, it remains unknown how to generate effective xenoantigen-specific Tr1 cells in vitro from naive CD4^+^ T cells.

Here, we describe a reliable strategy to induce and expand IL-10-secreting xenoantigen-specific human Tr1 cells in vitro, which may allow a more efficient strategy in transplantation immunotherapy.

## 2. Materials and Methods

### 2.1. Isolation of PBMC and Human CD4^+^ T Cells

Human PBMC samples came from the peripheral blood of two male and two female volunteers aged 28–58 years by using lymphocyte separation solution (TBD, Tianjin, China). According to the manufacturer's protocol, the naive CD4^+^ T Cell Isolation Kit (StemCell Technologies, Vancouver, BC, Canada) was used to sort CD4^+^ T cells from freshly isolated human PBMCs. Then, the lymphocyte separation solution (TBD, Tianjin, China) was used to isolate porcine PBMCs from the heparinized peripheral blood of adult landrace pigs. The porcine PBMCs were used as xenogeneic stimulator cells. All experiments in this study were approved by the Medical Ethics Committee and Animal Research Ethics Communities of Sichuan University. All volunteers signed an informed consent form.

### 2.2. Expansion of Human Tr1 Cells Stimulated with Xenoantigen In Vitro

Functional human Tr1 cells with xenoantigen specificity (XN-1) were generated in a coculture system of CD4^+^ T cells and irradiated (30 Gy) porcine PBMCs (xenogeneic PBMC: CD4^+^ T cells, 4 : 1) in RPMI 1640 medium at 37°C and 5% CO_2_ in 96-well U-bottom plates (BD Biosciences, Franklin Lakes, NJ, USA) for seven days as one cycle of xenoantigen stimulation. The coculture system was supplemented with 10% human AB serum, 2 mM glutamine, 25 mM hydroxyethyl piperazineethanesulfonic acid (HEPES), 50 U/ml penicillin, 50 mg/ml streptomycin (all bought from Gibco; Thermo Fisher Scientific, Inc.), and 50 mM 2-mercaptoethanol (2-ME) (Sigma; Merck KGaA, Darmstadt, Germany) in the presence of recombinant human IL-10 (10 ng/ml, ProSpec-Tany TechnoGene Ltd., East Brunswick, NJ, USA), recombinant human IL-15 (5 ng/ml, ProSpec-Tany TechnoGene Ltd.), IL-2 (40 U/ml) (Chiron, Emeryville, CA, USA), and Human T-Activator CD3/CD28 beads (Invitrogen, Carlsbad, CA, USA). The XN-1 cells were harvested after two subsequent cycles of xenoantigen stimulation. CD4^+^ T cells expanded as described above without pig PBMCs and IL-10 or only without pig PBMC after two subsequent cycles were used as polyclonal CD4^+^ Tr1 cells (PC-1) or polyclonally expanded Treg (CD4^+^ T cell), respectively.

### 2.3. Flow Cytometry

Cells were stained with fluorochrome-labeled human antigens CD4, CD39, CD49b, LAG-3, CD45RA, CD45RO, ICOS, and HLA-DR. All surface antibodies were from BD Biosciences. After 30 min of incubation at 4°C, cells were fixed in PBS containing 1.6% methanol-free formaldehyde (BD Biosciences). Intracellular staining was performed using fluorescently labeled anti-cytotoxic T-lymphocyte antigen-4 (CTLA-4) and FOXP3 antibodies (BD Biosciences). Cell samples and compensation beads were acquired using an LSRII flow cytometer (BD Biosciences).

### 2.4. RNA Extraction, Reverse Transcription of RNA, and RT-qPCR

Total RNA was extracted from Tr1 cells using TRIzol (Thermo Fisher Scientific, Inc.). According to the manufacturer's protocols, the reverse transcription of RNA into cDNA was performed through the Prime Script™ first-strand cDNA synthesis kit (Takara Bio, Dalian, China). The resulting cDNA was subjected to a real-time quantitative polymerase chain reaction (RT-qPCR) with Power SYBR Green PCR Master Mix (Applied Biosystems) on the Bio-Rad CFX Connect Real-Time System (Bio-Rad Laboratories, Inc., Hercules, CA, USA). The primers used are shown in Table 1. *GAPDH* normalized target gene expression as an internal reference gene used in this study [19].

### 2.5. Cytokine Analysis by the Enzyme-Linked Immunosorbent Assay (ELISA)

The supernatants of cell culture were collected after centrifugation at 3,000 rpm for 20 min to assess IL-10 secretion through the corresponding human ELISA kit (Human IL-10 ELISA Ready-SET-Go Kits; eBioscience) according to the manufacturer's instructions. The quantification of all samples followed a standard curve with standards containing known concentrations of recombinant protein.

### 2.6. Tr1 Cell Suppression Assay

The suppressive capacity of Tr1 cells in vitro was measured by a mixed lymphocyte reaction (MLR) assay. After labeling with 5 *μ*M 5,6-carboxyfluorescein diacetate succinimidyl ester (CFSE; Invitrogen), CFSE-labeled human PBMCs were incubated with 5 *μ*g/ml anti-human CD3 mAb and 2 *μ*g/ml anti-human CD28 mAb (BD Pharmingen) in RPMI 1640 medium (Invitrogen) containing 10% human AB serum. Irradiated (30 Gy) xenogeneic PBMCs or polyclonally expanded Tr1 cells or xenoantigen-expanded Tr1 cells were added to MLR cultures at 1/1, 1/2, and 1/16 dilutions. After seven days, the cultures were harvested to analyze the suppression capacity of Tr1 cells.

In the coculture system, 20 *μ*mol/l CD39 activity inhibitor polyoxometalate-1 (POM-1; Santa Cruz Biotechnology) was added into the MLR to evaluate the effect of CD39 on Treg-mediated suppression.

The proliferation of PBMCs was assessed depending on the percent-proliferating PBMCs cultured in the absence and presence of Tr1 cells. The percent proliferation of PBMCs in the absence of Tr1 cells was recognized as 100% of proliferation and 0% of suppression. Percent suppression of proliferating PBMCs was determined as %suppression = (percent‐proliferating PBMCs in the presence of Tr1/percent‐proliferating PBMCs) × 100%.

### 2.7. Statistical Analysis

Student's *t*-test (two-tailed) was performed to analyze the difference across two groups. One-way analysis of variance with Tukey's multiple comparison test was used to test the mean difference involving multiple groups by using SPSS version 20 (IBM Corp., Armonk, NY, USA). The data were summarized as means ± standard; *P* < 0.05 was considered statistically significant.

## 3. Results

### 3.1. Xenoantigen Stimulation Does Not Affect Tr1 Cell Expansion

After seven days of Tr1 cell expansion with different antigens, the average expansion fold of CD4^+^ T cells, polyclonally stimulated Tr1 cells (PC-1), and xenoantigen-stimulated Tr1 cells (XN-1) cells was 2.36 ± 0.67, 2.42 ± 0.80, and 3.07 ± 0.55, respectively. The CD4^+^ T, PC-1, and XN-1 cell expansion after 14 days of antigen stimulation was significantly increased (CD4^+^ T expansion fold: 42.38 ± 18.41, PC-1 expansion fold: 44.72 ± 10.42, and XN-1 expansion fold: 47.34 ± 17.19). There were no significant expansion changes among CD4^+^ T, PC-1, and XN-1 cells (Figure 1(c)). These data showed that xenoantigen stimulation did not affect the expansion of Tr1 cells in vitro.

### 3.2. Tr1 Cells Expanded with Xenoantigen Stimulation Acquire an Activated Treg Phenotype

After 14 days of xenoantigen or polyclonal stimulation, the Tr1 cell phenotype was examined by flow cytometry. XN-1 expressed a higher level CD49b and LAG-3 (73.5%; 74.5%) than PC-1 (68.5%; 71.3%) and CD4^+^ cells (43.5%; 43.7%). Moreover, both XN-1 and PC-1 expressed high levels of CTLA-4 and ICOS but no expression of FOXP3. After two subsequent cycles of stimulation, XN-1 expressed more HLA-DR (62.1%) than PC-1 (43.3%) and CD4^+^ T cells (58.3%). Interestingly, XN-1 expressed high levels of CD39 (73.8% of xenoantigen stimulation), which is characterized as a functional marker of Tregs. Meanwhile, Tr1 cells expressed the effector memory Treg phenotype both on cells expanded with xenoantigen stimulation or polyclonal stimulation, characterized by a high level of CD45RO but a low level of CCR7. In XN-1 cells, CD45RO^+^CCR7^−^ cells expressed a higher level of CD39 (71.5%) than PC-1 cells (Figures 1(a) and 1(b)). These results demonstrated that XN-1 showed the effector memory Treg phenotype, and CD39 might play an important role in XN-1 cells.

RT-qPCR results showed that XN-1 and PC-1 cells highly expressed IL-10, respectively, at levels 3.15 ± 0.25-fold and 7.93 ± 0.49-fold higher than CD4^+^ T cells, after two cycles of stimulation. However, XN-1 cells showed more IL-10 expression than PC-1 cells (*P* < 0.01). Moreover, the expression of IL-5 in PC-1 and XN-1 cells was 2.53 ± 0.11- and 5.77 ± 0.27-fold higher than that in CD4^+^ T cells. The IL-5 expression in XN-1 cells was significantly higher compared to that in PC-1 cells (*P* < 0.01). XN-1 cells showed a slightly elevated expression of Tr1 cell functional genes, TGF-*β*, and GITR compared to PC-1 cells (Figure 2(a)).

We then measured the IL-10 secretion in culture supernatants of Tr1 cells with two subsequence cycles of xenoantigen- or polyclonally stimulated expansion. IL-10 concentration of XN-1 cells was 198.50 ± 19.45 pg/ml, which was significantly higher than the 132.63 ± 4.78 pg/ml level of PC-1 cells (*P* < 0.05) (Figure 2(b)). These results demonstrated that Tr1 cells could secrete a large amount of IL-10 after xenoantigen stimulation.

After two subsequent antigen stimulation cycles, cells were harvested to detect the TCR V*β* family's gene expression. The increased expression of TCR V*β*2, TCR V*β*9, and TCR V*β*13 was observed after antigen stimulation. Also, the expression of TCR V*β*2, TCR V*β*9, and TCR V*β*13 was higher in XN-1 than in PC-1 cells (Figure 2(c)). These results indicated that XN-1 cells recognize xenoantigens via TCR V*β*2, TCR V*β*9, and TCR V*β*13.

### 3.3. IL-5 Can Affect Tr1 Cell Proliferation but Not Its Phenotype Expression

TPC-1 and XN-1 cells were stimulated with polyclonal stimulation in the presence of the anti-IL-5 antibody (PC-1+anti-IL-5) or xenoantigen stimulation in the presence of the anti-IL-5 antibody (XN-1+anti-IL-5), respectively, to assess the effect of IL-5 on Tr1 cell induction. In the result of trypan blue exclusion, after seven days of Tr1 cell expansion, the average expansion fold of PC-1, PC-1+anti-IL-5, XN-1, and XN-1+anti-IL-5 was 3.25 ± 1.77, 1.96 ± 0.28, 2.88 ± 1.24, and 1.80 ± 0.07, respectively, and there were no significant changes among the four groups. After 14 days of Tr1 cell expansion, the average expansion fold of PC-1+anti-IL-5 and XN-1+anti-IL-5 was significantly lower than the expansion of PC-1 and XN-1 (*P* < 0.01) (Figure 3(a)).

Then, we detected the phenotypic characteristics of Tr1 cell expansion with an anti-IL-5 antibody by flow cytometry. After two cycles of antigen expansion, PC-1+anti-IL-5 and XN-1+anti-IL-5 expressed slightly low CD49b and LAG-3 compared with PC-1 and XN-1. In contrast, both PC-1+anti-IL-5 and XN-1+anti-IL-5 expressed higher HLA-DR and ICOS levels compared with PC-1 and XN-1, respectively. The addition of anti-IL-5 antibodies made no difference to the activation of PC-1 and XN-1 cells. HLA-DR and ICOS were still highly expressed (Figure 4). Meanwhile, anti-IL-5 antibodies did not affect PC-1 and XN-1 cell expression of CTLA-4 and IL-10, which retained low expression or no expression of FOXP3 and IL-4 (Figure 4). The results indicated that IL-5 affects the proliferation of PC-1 and XN-1 cells but without changes to their phenotypic characteristics.

### 3.4. Xenoantigen-Stimulated Tr1 Cells Enhanced Suppressive Capacity via CD39

XN-1 cells were stimulated with xenoantigen in the presence of the CD39 inhibitor POM-1, and a Xeno MLR assay measured the suppressive function to examine the effect of CD39 on XN-1. XN-1 with POM-1 exhibited a lower xenoantigen-specific suppressive capacity than XN-1 cells, as evidenced by 73.89% ± 6.72% and 91.81% ± 3.50% suppression at high responder cell : Tr1 ratios of 1 : 1. XN-1 with POM-1 exhibited a significantly lower xenoantigen-specific suppressive capacity than XN-1 at low responder cell : Tr1 ratios of 1 : 1/2 (*P* < 0.01) and 1 : 1/16 (*P* < 0.01), respectively (Figure 3(b)). The results indicated that xenoantigen-stimulated Tr1 cells acquire an enhanced suppressive capacity via CD39.

## 4. Discussion

The tremendous challenges for clinical therapeutic application of antigen-specific Tregs have been how to solve the insufficient number of cells and find an effective way to expand Tregs. Antigen-specific Tregs with highly suppressive properties may mitigate systemic immunosuppression risk and minimize Tregs' requirement for cellar therapy ([20]; Ma et al., 2016). Various experimental conditions have been investigated by in vitro studies for large-scale expansion of antigen-specific Tregs [21–23]. In this study, a feasible and straightforward strategy using two cycles of xenoantigen stimulation with recombinant human IL-10 was developed to expand xenoantigen-specific human Tr1 cells selectively. Our results show that by applying this method, xenoantigen stimulation exerts no influence on the expansion of Tr1 cells in vitro but activated the functional Treg phenotype.

IL-10 is involved in modulating Treg-mediated suppression of xenogeneic responses. A previous in vitro study has revealed that IL-10 polarized naive CD4^+^ T cells toward Tr1-like T cells, secreting a higher level of IL-10 [24]. Numerous studies showed that antigen-specific Tr1 cells produced a high level of IL-10 and suppressed immune responses [25, 26]. In this research, the secretion and gene expression of IL-10 produced by XN-1 cells were significantly higher than those produced by PC-l cells. Therefore, these results indicated that xenoantigen stimulation promotes the Tr1 cells to secrete IL-10 and enhances the suppressive function of Tr1 cells. In our study, we found that XN-1 cells upregulated the expression of IL-5. A previous study showed that IL-5 promoted the expansion of autoantigen-specific Tregs and maintained alloantigen-specific tolerance [27]. However, the effect of IL-5 on the IL-10-induced Tr1 cells remained unclear. Interestingly, here we found that anti-IL-5 reduced PC-1 and XN-1 cell expansion but did not affect their phenotype. The results indicated that IL-5 is closely related to the expansion of antigen-specific Tr1 cells.

Tr1 cells exhibit restricted TCR V*β* families following xenoantigen stimulation [24]. The activation of Treg cells' suppressive function is related to the availability of antigen and the affinity of TCRs or the recognized antigens [28]. This study identified a higher expression of TCR V*β*2, TCR V*β*9, and TCR V*β*13 in XN-1 than in PC-1. These results indicated that xenoantigen-specific Tr1 cells recognized xenoantigen via specific repertoires in TCR V*β* families to exert regulatory functions.

Additionally, xenoantigen-specific Tr1 cells were obtained with only two cycles of expansion. XN-1 cells can express a high level of CD45RO but without CCR7, which has been identified as an effector marker of effector memory T cells [29]. Surprisingly, a high expression of CD45RO^+^CCR7^−^ cells was found in XN-Tr1 cells, with a high level of CD39. CD39 is an integral vascular and immune ectonucleotidase critical to maintaining homeostasis and regulating the immune response. A study showed that the level of expression and activity of CD39 in Treg cells directly modulates their immunosuppressive capacity via the generation of adenosine [30].

Consequently, we hypothesized that the xenoantigen-stimulated Tr1 cells enhanced suppressive capacity via CD39. In this study, the xenoantigen stimulation (XN-1) in the presence of the CD39 inhibitor POM-1 showed decreased PBMC proliferation inhibition in a dose-dependent manner, suggesting that xenoantigen-stimulated Tr1 cells demonstrated an enhanced suppressive capacity via CD39. However, the mechanisms underlying CD39 involved in the suppressive function of human xenoantigen-specific Tregs remain largely unknown. Further research is needed to explore how CD39 enhanced suppressive capacity in human xenoantigen-specific regulatory T cells.

## 5. Conclusion

In conclusion, we described an effective and feasible protocol to obtain large amount of xenoantigen-specific human Tr1 cells. This study demonstrated that xenoantigen-stimulated Tr1 cells recognized xenoantigen via specific repertoires in TCR V*β* families to exert a regulatory function and displayed enhanced suppressive capacity via CD39, thus providing theoretical new insights into the modulating immune tolerance in clinical xenotransplantation.

## Figures and Tables

**Figure 1:** Treg expansion with xenoantigen or polyclonal stimulation and phenotypical characterization of expanded Tr1 cells. (a, b) The expression levels of CD49b, LAG-3, FOXP3, CCR7, CTLA-4, HLA-DR, ICOS, and CD39 by XN-1, PC-1, and CD4^+^ T cells are presented as the percentage of CD4^+^CD25^+^ with coexpressing individual molecules examined. PC-1: polyclonal Tr1 cells; XN-1: Tr1 cells with xenoantigen specificity. (c) The cell number of expanded CD4^+^ T, PC-1, and XN-1 cells was calculated after seven days and 14 days of polyclonal or xenoantigen stimulation. Treg expansion was determined as fold expansion, summarized as cell number of expanded Tr1 cells at the end of each stimulation cycle divided by the number of Tr1 cells at the beginning of expansion culture. Data are represented as mean ± SD of three individual experiments in dots.

**Figure 2:** Gene expression of Tr1 cells and suppressive capacity of expanded Tr1 cells with xenoantigen. (a) Gene expression of IL-10, IL-4, IL-2, TGF-*β*, GITR, and TCR family in PC-1, XN-1, and CD4+ cells. (b) IL-10 secretion by ELISA. (c) Gene expression of the TCR V*β* family. (d) Suppressive capacity of PC-1 and XN-1 cells in polyclonally stimulated MLR. (e) Suppressive capacity of PC-1 and XN-1 cells in allogenic stimulated MLR. (f) Suppressive capacity of PC-1 and XN-1 cells in xenoantigen-driven stimulated MLR. PC-1: polyclonal Tr1; XN-1: Tr1with xenoantigen specificity. ^∗^*P* < 0.05; ^∗∗^*P* < 0.01.

**Figure 3:** Tr1 expansion in the presence of the anti-IL-5 antibody and suppressive capacity of expanded XN-1 cells with POM-1. (a) PC-1 and XN-1 cells were counted after 7 days and 14 days of polyclonal or xenoantigen stimulation. Tr1 expansion efficacy was determined as fold expansion as mentioned in Figure 1. (b) XN-1+POM-1, PC-1, and XN-1 cell suppression of responder cell proliferation in xenoantigen-driven stimulated MLR. PC-1: polyclonal Tr1; XN-1+POM-1: Tr1 with xenoantigen specificity in the presence of the CD39 inhibitor POM-1; XN-1: Tr1 with xenoantigen specificity. ^∗^*P* < 0.05; ^∗∗^*P* < 0.01.

**Figure 4:** Phenotypic characterization of expanded Tr1 cells with xenoantigen or polyclonal stimulation in the presence of anti-IL-5 antibodies.

**Table 1:** Sequence of primers in this study.

Gene	Sequence
IL10 sense	5′-GCC TAA CAT GCT TCG AGA TC-3′
IL10 antisense	5′-TGA TGT CTG GGT CTT GGT TC-3′
PD-1 sense	5′-TTTCAGGAATGGGTTCCAAG-3′
PD-1 antisense	5′-ACATCCTACGGTCCCAAGGT-3′
IL2 sense	5′-GAACTAAAGGGATCTGAAACAACATTC-3′
IL2 antisense	5′-TGTTGAGATGATGCTTTGACAAAA-3′
IL4 sense	5′-AGAAGACTCTGTGCACCGAGTTGA-3′
IL4 antisense	5′-CTCTCATGATCGTCTTTAGCCTTT-3′
IFN-gamma sense	5′-GGC ATT TTG AAG AAT TGG AAA G-3′
IFN-gamma antisense	5′-TTT GGA TGC TCT GGT CAT CTT-3′
TGF-beta sense	5′-TGGAAACCCACAACGAAATC-3′
TGF-beta antisense	5′-GGGTTCAGGTACCGCTTCTC-3′
IL-5 sense	5′-GGCACTGCTTTCTACTCATCGA-3′
IL-5 antisense	5′-AGTTGGTGATTTTTATGTACAGGAACA-3′
GITR sense	5′-GTTTTGGCTTCCAGTGTATCGA-3′
GITR antisense	5′-AACACAGTGAGAAACCCGAACT-3′
GAPDH sense	5′-TGCACCACCAACTGCTTAGC-3′
GAPDH antisense	5′-GGCATGGACTGTGGTCATGAG-3′

## Data Availability

The data used during the present study are available from the corresponding author upon reasonable request.
